The article "The Hair Growth-Promoting Effect of Gardenia florida Fruit Extract and Its Molecular Regulation" was published in 2022. Journal: Evid Based Complement Alternat Med.

# The Hair Growth-Promoting Effect of *Gardenia florida* Fruit Extract and Its Molecular Regulation

**DOI:** 10.1155/2022/8498974

**Published:** 2022-09-19

**Authors:** Xiaojin Liu, Tiancheng Ji, Haoya Hu, Xiaobing Lv, Guoping Zhu

**Affiliations:** Anhui Provincial Key Laboratory of Molecular Enzymology and Mechanism of Major Diseases, College of Life Sciences, Anhui Normal University, Wuhu, China

## Abstract

As a herbal medicine, the extract from the fruits of *Gardenia florida* has been widely used for its antioxidative, hypoglycemic, and anti-inflammatory properties. However, whether *G. florida* fruit extract (GFFE) regulates hair growth has been rarely studied. This study was the first application of GFFE on hair growth both in vitro (human dermal papilla cells, hDPCs) and in vivo (C57BL/6 mice). The effects of GFFE on cell proliferation and hair growth-associated gene expression in hDPCs were examined. Moreover, GFFE was applied topically on the hair-shaved skin of male C57BL/6 mice, the hair length was measured, and the skin histological profile was investigated. GFFE promoted the proliferation of hDPCs and significantly stimulated hair growth-promoting genes, including vascular endothelial growth factor (VEGF) and Wnt/*β*-catenin signals, but suppressed the expression of the hair loss-related gene transforming growth factor-*β*1 (TGF-*β*). Furthermore, GFFE treatment resulted in a significant increase in the number, size, and depth of cultured hair follicles and stimulated the growth of hair with local effects in mice. In summary, the results provided the preclinical data to support the much potential use of the natural product GFFE as a promising agent for hair growth.

## 1. Introduction

Recently, the number of hair loss patients has continued to increase, with a trend in younger people and females [1, 2]. Hair loss can occur because of heredity, accompanying comorbidity conditions, hormonal clutters, immune systems, nutritional scatters, environmental elements, mental disorders, and aging [3]. There are two most common forms of hair loss: alopecia areata (AA) and androgenetic alopecia (AGA) [4, 5]. In clinical, AA is caused by an autoimmune reaction, whereas AGA is the most frequent category of hair loss in men, which is defined as the result of the high sensitivity of scalp follicles to dihydrotestosterone (DHT) [6, 7].

HDPCs play key roles in the proliferation, differentiation, and hair cycle control of hair follicles [8]. Several genetic factors are discovered to be associated with the hair cycle and hair growth in DPCs, and mechanisms involving IGF-1 [9, 10], VEGF [11–13], epidermal growth factor (EGF) [14, 15], FGF-2 [16], endothelial nitric oxide synthase (eNOS) [4, 17], Wnt/*β*-catenin signaling pathway [18–20], prostaglandin E (PGE) [21], and prostaglandin F (PGF) [22] stimulate hair growth; however, the mechanism engaging 5*α*-reductase [23–26], TGF-*β* [17], FGF-5 [27], and prostaglandin D2 (PGD2) [28] are known to inhibit hair growth.

The article "The Hair Growth-Promoting Effect of Gardenia florida Fruit Extract and Its Molecular Regulation" was published in 2022. Journal: Evid Based Complement Alternat Med.

Hair loss is recognized as a common dermatological problem, which significantly influences the patient quality of life and mental state, and the development of treatment agents has been markedly growing. Current drugs available for hair loss treatment include medications such as Minoxidil® and Finasteride® [29, 30]. Minoxidil is proven to promote hair growth as a vasodilator to deliver nutrients and oxygen to the hair follicle, thereby increasing hypertrichosis, and has adverse systemic effects such as myocardial and anorexia infarction [31, 32]. Finasteride associated with adverse sexual effects is developed as a competitive inhibitor of type II 5*α*-reductase and is not valid for women [33, 34].

Therefore, the development of new ways to enhance hair growth and prevent hair loss is urgently needed in the hair care industry [35, 36]. Recently, many herbal topical formulations are available on the market, with many advantages such as natural substances, high safety, low-cost, patient compliance, the concept of treatment plus recuperation, and multi-target onset for hair growth promotion or hair loss treatment [35, 37, 38].

As a traditional herbal medicine that is widely distributed in most parts of China, *Gardenia florida* fruits have been used in antioxidative, anti-inflammatory, and hypoglycemic purposes [39]. This study innovatively presents the first application of GFFE in the field of hair growth and explores the mechanism of action: we demonstrated that GFFE had the potential to enhance hDPCs proliferation in a dose-dependent manner. Furthermore, we evaluated the hair growth-related genes, and the results showed that TGF-*β*1 and DKK1 decreased; however, the LEF1, Wnt5a, *β*-catenin, and VEGF increased; we also verified the effects of GFFE treatment on protein expression of TGF-*β*1, Wnt5a, and VEGF in hDPCs by western blot examination. Then, we investigated GFFE for its potential effect in the C57BL/6 mouse model showing the hair length difference, and histological findings verified that retardation of entry into catagen occurred in response to GFFE application. Taken together, these data considered that GFFE may be a new ingredient for hair growth-promoting and hair loss treatment potential.

## 2. Materials and Methods

### 2.1. Reagent

*G. florida* fruit extract (GFFE) was purchased from the Nanjing DASF Biotechnology Co., Ltd (Nanjing, China). Human dermal papilla cells (hDPCs) were purchased from Sciencell Research Laboratories, Inc.

The article "The Hair Growth-Promoting Effect of Gardenia florida Fruit Extract and Its Molecular Regulation" was published in 2022. Journal: Evid Based Complement Alternat Med.

### 2.2. Cell Proliferation Test

Cell proliferation was measured using Cell Counting Kit-8 (CCK-8, Shanghai Hanheng Biotechnology Co., Ltd., Shanghai, China). Human DP cells were seeded in 96-well plates at a density of 3,000 cells/well and incubated in a humidified atmosphere with air and 5% CO_2_ at 37°C. Cultured cells were then treated with various concentrations of GFFE for 24 hours according to the kit protocol. CCK-8 solution was added, followed by a 4-hour incubation, and absorbance at 450 nm was measured on a TECAN Enzyme standard instrument Spark 10 M. The cell proliferation rates were calculated from OD and represented as percentages of negative control (NC).

### 2.3. RNA Extraction and Real-Time PCR Quantitative Reverse Transcription PCR

In vitro model, hDPCs were plated on a 6-well plate (1.0 × 10^5^) and incubated until grown to 80–90% confluence in a 10% FBS DMEM medium. After culture with serum-free DMEM medium for 24 h, the cells were added to each treatment and incubated for 24 h in aserum-free DMEM (NC), with 19.5 *μ*g/mL of GFFE. Total RNA was extracted using Monzol™ Reagent (Monad Biotech Co., Ltd, China) according to the manufacturer's instructions. Glyceraldehyde 3-phosphate dehydrogenase (GAPDH) was used as an internal reference. For RT-PCR, 1 *µ*l each of the forward primer (10 ng/*µ*l) and reverse primer (10 ng/*µ*l) per well, iTaq universal Green supermix (2x) 10 *µ*l, nuclease-free H_2_O 6 *µ*l, and cDNA 2 *µ*l were mixed to a final volume of 20 *µ*l. The PCR procedure software recorded the average fluorescence value of each cycle of the reaction. The relative expression levels of different genes in the cells were obtained by comparing the Ct values. The experiment was repeated three times with three replicates seated per reaction.

As for qRT-PCR, MonAmpTM ChemoHS qPCR Mix (Monad Biotech Co., Ltd, China) was used following the instructions of the manufacturer. The qRT-PCR was performed using a BIO-RAD CFX96^TM^ Real-Time PCR system (BIO-RAD, USA) with the following setting condition: 95°C for 10 min; 40 cycles including 95°C for 10 sec, 60°C for 30 sec, and 72°C for 30 sec. cDNA was amplified using MonScript™ RTIII All-in-One Mix with dsDNase (Monad Biotech Co., Ltd, China).

Primers were used as follows: GAPDH, 5′-TGTTGCCATCAATGACCCCTT-3′ (forward), GAPDH, 5′-CTCCACGACGTACTCAGCG-3′ (reverse) [40]; VEGF, 5′-TCTTCAAGCCATCCTGTGTG-3′ (forward), VEGF, 5′-GCGAGTCTGTGTTTTTGCAG-3′ (reverse) [41]; Wnt5a, 5′-TTGAAGCCAATTCTTGGTGGTCGC-3′ (forward), Wnt5a 5′- TGGTCCTGATACAAGTGGCACAGT-3′ (reverse) [40]; TGF-*β*1, 5′-GCAGAAGGATCACCACAACC-3′ (forward), TGF-*β*1, 5′-TGTCTGCACTGCGGAGGTAT-3′ (reverse) [42]; DKK1, 5′-CCTTGAACTCGGTTCTCAATTCC-3′ (forward), DKK1, 5′-CAATGGTCTGGTACTTATTCCCG-3′ (reverse) [40]; *β*1-catenin, 5′-AACTTGCTCAGGACAAGGAA-3′ (forward), *β*1-catenin, 5′-TCCTAAAGGATGATTTACAGGTC-3′ (reverse) [42]; LEF1, 5′-GAATTAGCACGGAAAGAAAGA-3′ (forward), LEF1, 5′-ACCTGTACCTGATGCAGATT-3′ (reverse) [40].

The article "The Hair Growth-Promoting Effect of Gardenia florida Fruit Extract and Its Molecular Regulation" was published in 2022. Journal: Evid Based Complement Alternat Med.

### 2.4. Western Blot Analysis

The cultured cells were collected and lysed in RIPA buffer (Beyotime) with protease inhibitors (Beyotime) after rinsing twice with PBS (precooled at 4°C). Protein was quantified with a BCA protein concentration determination kit (Beyotime), and then separated by SDS- polyacrylamide gel electrophoresis and electroblotted onto polyvinylidene fluoride membranes. After blocking in 5% nonfat milk for 2 h at 25°C, the membranes were probed with primary antibodies followed by horseradish peroxidase-conjugated secondary antibodies (Proteintech Group, Inc.). Primary antibodies used were rabbit anti-VEGF protein (1 : 1000, Proteintech Group, Inc.), rabbit anti-Wnt5a (1 : 1000, Proteintech Group, Inc.), rabbit anti-TGF-*β*1 (1 : 1000, Proteintech Group, Inc.) and rabbit anti-Tubulin (l : 1000, Proteintech Group, Inc.). We used BeyoECL Star (Beyotime) reagent to detect protein.

### 2.5. Animals

The animals were housed in a temperature-controlled room with a 12-h light/dark cycle and were allowed free access to food and water in the course of experiments. Twenty-five male five-week-old C57BL/6 mice (Henan Sikebas Biotechnology Co., Ltd., China) in 5 randomized groups (*n* = 5) were used for this study. The dorsal area hairs (approximately 2 cm in width and 3 cm in length) on the back of the mouse in the telogen phase were shaved 24 h before applying the treatments. Animals in group 1 served as NC (water), and group 2 received 2% minoxidil as a positive control group. The animals in group 3, group 4, and group 5 received different doses (0.5%, 1.0%, and 2.0%) of GFFE, respectively. The 5 groups were applied topically to the test area with 0.2 mL once a day, for 30 days. The animals were isolated for an hour and then kept back in their respective cages. During the application period, differences between treatment and nontreatment groups in average body weight or abnormalities in the mice were not observed. The hair regrowth activities of GFFE were evaluated by observing and photographing the back skin of mice. On day 14, day 21, and day 30, 10 hairs were plucked from the mice's shaved area randomly from all groups and the average length of each treatment was measured.

### 2.6. Histopathology of Hair Growth

Dorsal skin tissues from each mouse were excised and fixed in 4% neutral formalin for 24 h. They were embedded in paraffin after routine tissue processing. For the hair follicle's histopathologic evaluation, a 4 *μ*m tissue section was stained with the standard hematoxylin and eosin (H&E staining) protocol [43]. Hematoxylin is a basic dye that stains nucleic acids purplish blue; eosin is an acidic dye that stains cytoplasm and extracellular matrix pink. The morphology and the number of hair follicles were evaluated by veterinary pathologists.

The article "The Hair Growth-Promoting Effect of Gardenia florida Fruit Extract and Its Molecular Regulation" was published in 2022. Journal: Evid Based Complement Alternat Med.

### 2.7. Hair Length Determination

On 14, 21, and 30 days after beginning the animal experiment, 10 hairs were plucked from the mice's shaved area randomly from all groups and the average length of each treatment was measured.

### 2.8. Statistical Analysis

All treatments were repeated at least three times. Data represent biological replicates. The data were statistically analyzed by Student's *t*-test for the comparison among groups using SPSS WIN (v25.0). The results were considered statistically significant if the *p* values were less than 0.05.

## 3. Results

### 3.1. Cell Proliferation Assays of GFFE

Dose-dependent proliferative effects of GFFE (0.008%, 0.016%, 0.032%) tested on hDPCS were first examined by CCK-8 assay following 4-h culture (Figure 1). After incubation for 48 hours, the number of expanded hDPCs was efficiently greater in all GFFE groups than in the NC (0%), reaching 106.78% (^*∗*^), 110.67% (^*∗*^), and 112.92% (^*∗∗*^), respectively. Particularly, the 0.032% GFFE exhibited the highest cell proliferation rates than the NC group. Collectively, these results suggest that GFFE facilitates the proliferation of DPCs and improves the hair-inducing abilities of these cells.

### 3.2. Comparison of Wnt/*β*-Catenin, VEFG, and TGF-*β*1 Signaling mRNA Expression

Wnt signals play a crucial role in the activation of bulge stem cells to progress toward hair formation and the induction of the anagen phase in hair growth which is required for the establishment of the hair follicle [44]. The Wnts comprise a large class of secreted proteins. *β*-Catenin, the transducer of Wnt signaling, has been reported to contribute to the maintenance of HF structures and is translocated to the nucleus which is important for the development and growth of hair follicles [45]. It was reported that transgenic overexpression of LEF1 leads to regrowth of hair follicle formation in the epidermis [46]. As a specific endogenous Wnt antagonist, DKK1 decreased hair follicle sizes by blocking the activation of Wnt signaling [47]. DKK1 was also reported to promote hair follicle regression [18, 48]. Wnt5*a*, which has been classified as a noncanonical Wnt family member, can also activate *β*-catenin signaling in the presence of the appropriate Frizzled receptor 4 [49]. Genes responsible for Wnt/*β*-catenin signaling including DKK1, LEF1, Wnt5*a*, and *β*-catenin mRNA were investigated by means of RT-PCR.

The article "The Hair Growth-Promoting Effect of Gardenia florida Fruit Extract and Its Molecular Regulation" was published in 2022. Journal: Evid Based Complement Alternat Med.

We found the mRNA level of Dkk1, a negative regulator of Wnt/*β*-catenin signaling, was reduced by 21%, 54%, and 67% in hDPCs treated with 0.008%, 0.016%, and 0.032% GFFE, respectively; the mRNA level of LEF1, a positive regulator of Wnt/*β*-catenin signaling, was increased by 66% (^*∗∗*^), 22% (^*∗*^), and 25% (^*∗*^) in hDPCs treated with 0.008%, 0.016%, and 0.032% GFFE, respectively; the mRNA level of *wnt5a*, a positive regulator of Wnt/*β*-catenin signaling, was increased by 162% (^*∗∗*^), 36% (^*∗∗*^), and 5% (no statistically significant differences) in hDPCs treated with 0.008%, 0.016%, and 0.032% GFFE, respectively; the mRNA level of *β-catenin*, a positive regulator of Wnt/*β*-catenin signaling, was increased by 32% and 91% in hDPCs treated with 0.16% and 0.032% GFFE, respectively, but 0.008% GFFE decreased the expression of *β-catenin* (^*∗∗*^) (Figure 2).

DHT was described to stimulate the synthesis of TGF-*β*2 in DPCs, and these sequential events contributed to the shortening of the human hair cycle [50], [56]. Androgen-inducible TGF-*β*1 was regarded to regulate hair growth suppression by dose-dependently repressed hDPCs growth [17], [57]. However, TGF-*β* antagonists were effective in preventing catagen-like morphological changes and promoting elongation of hair follicles. In this study, GFFE decreased the expression of TGF-*β*1 in hDPCs. 0.008%, 0.016%, and 0.032% GFFE treatments showed 57%, 41%, and 64% decrease in TGF-*β*1 mRNA expression compared to NC, respectively (^*∗∗*^) (Figure 2).

Growth factor VEGF stimulates hair growth by increasing the base of the follicle diameter and supply of nutrients to the hair follicle [4]. It was demonstrated that the highest expression of VEGF was found in fibrous sheath fibroblasts and dermal fibroblasts in hDPCs [51]. However, the highest expression of *VEGF* mRNA is in the anagen phase and it is less expressed in the catagen and telogen phases in DPCs during the hair growth cycle [52]. In this study, 0.008% and 0.016% GFFE showed 68% (^*∗∗*^) and 19% (^*∗*^) greater *VEGF* mRNA expression compared to NC, respectively. However, 0.032% GFFE showed 6% (no statistically significant differences) decreased *VEGF* mRNA expression compared to NC (Figure 2).

We treated cultured hDPCs with different concentrations of GFFE (0, 0.008%, 0.016%, and 0.032%) to determine whether GFFE affects the hair-inducing ability of hDPCs. The above results suggested that GFFE could promote the hair-inducing ability of hDPCs. Next, we evaluated the effects of the GFFE on the protein expression and activity of Wnt5*a*, VEGF, and TGF-*β*1 by western blotting test.

The article "The Hair Growth-Promoting Effect of Gardenia florida Fruit Extract and Its Molecular Regulation" was published in 2022. Journal: Evid Based Complement Alternat Med.

### 3.3. Effects of the Protein Expression of Wnt5*α*, VEGF, and TGF-*β*1-Related Molecules in GFFE-Treated hDPCs

In hDPCs, the immunoblot analysis showed that the active Wnt5*a* protein level increased with all GFFE treatment groups. 0.008%, 0.016%, and 0.32% GFFE groups showed 66% (^*∗∗*^), 79% (^*∗∗*^), and 25% (^*∗*^) greater Wnt5*a* protein expression than NC, respectively (Figure 3(a)). The active TGF-*β*1 protein level decreased in hDPCs treated with all GFFE treatment groups; 0.008%, 0.016%, and 0.032% GFFE groups showed 6% (no significant statistical differences), 67% (^*∗∗*^), and 81% (^*∗∗*^) attenuated TGF-*β*1 protein expression compared to NC, respectively (Figure 3(b)). However, the results suggested that GFFE induced VEGF activation in a dose-dependent manner. 0.032% GFFE groups showed 76% (^*∗∗*^) increased VEGF protein level compared to NC, but VEGF protein level with 0.008% and 0.016% GFFE treatments showed 24% (^*∗∗*^) and 18% (^*∗*^) decreased level compared to NC, respectively (Figure 3(c)). More research is needed to explain it. In summary, the mechanism of GFFE promoting the proliferation of hDPCs in vitro may be related to the Wnt/*β*-catenin signaling pathway, TGF-*β*1 factor regulation, and VEGF factor regulation. However, there are still many mechanisms involved in hair growth and DPC proliferation, and many other related factors should be studied in the Wnt/*β*-catenin signaling pathway. Therefore, the detailed mechanism of GFFE promoting the growth and proliferation of hDPCs in vivo needs to be further studied.

### 3.4. Hair Regeneration Was Induced by Topical Treatment with GFFE

Here, we used a commonly used in vivo C57BL/6J mouse dorsal skin model to test whether GFFE can increase hair regeneration. Male mice at 44 days of age (telogen) were shaved on the back when dorsal skin hair follicles are in telogen. GFFE or NC treatment was applied topically every day. In NC mice, only a few scattered pigmented spots were apparent at least until day 21. In contrast, both the GFEE (0.5%, 1.0%, and 2.0%) and 2% Minoxidil groups achieved hair regrowth and became remarkably grey after 7 days (Figure 4). Formation and differentiation of hair follicles in GFFE-treated mice were correspondingly demonstrated by histological analyses.

### 3.5. Histopathology of Depilated Mice

The morphology of the hair follicles was evaluated histologically to define the effect of GFFE on hair growth. The comparison and difference between NC, MXD, and GFFE groups in number, size, and depth of follicle were observed by histological photos (qualitative analysis in Figure 5); however, the length of dorsal skin tissues hairs was evaluated by quantitative analysis in Figure 6. It was observed that the depth of the hair follicle was deeper, the dermal layers were thicker, and the length of the hair follicular shaft was longer in 1.0% (Figure 5(d)) and 2.0% (Figure 5(e)) GFFE group than those in NC (Figure 5(a)) and Minoxidil groups (Figure 5(b)). Taken together, these findings suggested that GFFE could contribute to maintaining the anagen phase and preventing entry into the catagen phase in the hair cycle.

The article "The Hair Growth-Promoting Effect of Gardenia florida Fruit Extract and Its Molecular Regulation" was published in 2022. Journal: Evid Based Complement Alternat Med.

### 3.6. Hair Length Determination

10 hair follicles were plucked from the mice's shaved area randomly from all groups, and the average length of each treatment was measured on day 14, day 21, and day 30. In day 14, the hair length of NC, MXD, 0.5% GFFE, 1% GFFE, and 2% GFFE was 2.43 mm, 4.12 mm (^*∗∗*^), 3.68 mm (^*∗*^), 4.18 mm (^*∗∗*^), and 3.96 mm (^*∗*^), respectively. In day 21, the hair length of NC, MXD, 0.5% GFFE, 1% GFFE, and 2% GFFE was 4.93 mm, 7.86 mm (^*∗∗∗*^), 6.74 mm (^*∗∗*^), 7.91 mm (^*∗∗∗*^), and 7.60 mm (^*∗∗∗*^), respectively. In day 30, the hair length of NC, MXD, 0.5% GFFE, 1% GFFE, and 2% GFFE was 8.11 mm, 11.05 mm (^*∗∗*^), 10.21 mm (^*∗*^), 11.13 mm (^*∗∗*^), and 10.83 mm (^*∗*^), respectively (Figure 6).

## 4. Conclusions

In this study, GFFE showed strong hair growth-promoting activity. GFFE a was natural compound and has many pharmacological and physiological activities [39]. The hair-growth-promoting activities of GFFE are recognized as novel anti-aging effects. In summary, we demonstrated that GFFE could induce VEGF and Wnt/*β*-catenin signaling pathway activity while attenuating TGF-*β*1 synthesis activity in hDPCs and also found that GFFE up-regulated the protein expressions of VEGF and *β*-catenin and downregulated TGF-*β*. Moreover, GFFE promoted hair regeneration and repair in mouse models. Collectively, our results unveil a novel functional role of GFFE and strongly imply that GFFE can be developed as a herbal medicine for the treatment of hair loss diseases. In a future study, we will explore the specific constituents of antiremoval factors in GFFE as well as conduct GFFE in vivo and clinical trials to elucidate their application potential.

## Figures and Tables

**Figure 1:** The proliferative effects of GFFE on hDPCs were incubated with different concentrations of GFFE as indicated. Cell viability was measured by the CCK-8 assay, and the proliferation index after 48 hours was determined. NC: negative control (DMEM medium); the hDPCs were treated with various concentrations of GFFE (0.008%, 0.016%, and 0.032%). Data are reported as mean +  SEM. Student's *t*-test was used to compare data. ^*∗*^*P* < 0.05; ^*∗∗*^*P* < 0.01.

The article "The Hair Growth-Promoting Effect of Gardenia florida Fruit Extract and Its Molecular Regulation" was published in 2022. Journal: Evid Based Complement Alternat Med.

**Figure 2:** Quantitative real-time polymerase chain reaction (RT-qPCR) for DKK1, LEF1, Wnt5a, *β*-catenin, TGF-*β*1, and VEGF in GFFE-treated hDPCs. The DPCs (3.0 × 10^4^ cells/well) were cultured in serum-free DMEM for 24 h and then treated with GFFE at concentrations of 0, 0.008%, 0.016%, and 0.032% for 24 h; ^*∗*^*p* < 0.05 and ^*∗∗*^*p* < 0.01, compared with NC.

**Figure 3:** Expression levels of Wnt5a, TGF-*β*1, and VEGF protein in DPCs under different concentrations of GFFE. ^*∗*^*p* < 0.05 and ^*∗∗*^*p* < 0.01, compared with the negative control.

**Figure 4:** Hair growth-stimulating effect of GFFE in an in vivo C57BL/6 male mice model. Mice were shaved on postnatal day 44 and topically treated with NC or GFFE (dissolved in water at 0.5%, 1.0%, and 2.0% final) every day over 30 days. Photographs shown were taken on day 0, 7, 14, 21, and 30 after treatment. Indicative of anagen induction by the treatment, melanin pigmentation in the skin of GFFE-treated animals became visible as early as day 7; NC mice did not show significant pigmentation for at least 21 days. However, all mice in NC, GFFE, or Minoxidil treatments exhibited almost overall hair growth on day 30.

**Figure 5:** Histological analysis of hair follicles factor expression. Microphotographs of skin tissue sections showing different on the C57BL/6 mice's back skin (H&E staining, 100x magnification). (a) NC: negative control of C57BL/6 mice skin treated with water, (b) PC: positive control, 2.0% Minoxidil, (c) GFFE: 0.5%, (d) GFFE: 1.0%, and (e) GFFE: 2.0%.

**Figure 6:** Effects of various treatments on hair length of C57BL/6 mice at 21^st^ day. Values are expressed as mean ± standard error of mean. ^*∗*^*P* < 0.05, ^*∗∗*^*P* < 0.01, and ^*∗∗*^*P* < 0.001 versus NC group.

## Data Availability

The datasets generated and/or analyzed during the current study are not publicly available due to confidential reasons but are available from the corresponding author upon reasonable request.
